The article "DNM1: A Prognostic Biomarker Associated with Immune Infiltration in Colon Cancer—A Study Based on TCGA Database" was retracted in 2024. Reasons: signs of a paper mill; suspected computer-generated content; unreliable results or conclusions; concerns about the data.

# DNM1: A Prognostic Biomarker Associated with Immune Infiltration in Colon Cancer—A Study Based on TCGA Database

**DOI:** 10.1155/2021/4896106

**Published:** 2021-11-30

**Authors:** Mingchao Hu, Jianchun Gu, Wenzhao Su, Zhenjie Zhang, Baosong Zhu, Qiang Wang, Chungen Xing

**Affiliations:** ^1^Department of Gastrointestinal Surgery, The Second Affiliated Hospital of Soochow University, Suzhou 215000, China; ^2^Department of General Surgery, The Affiliated Jiangsu Shengze Hospital of Nanjing Medical University, Suzhou 215228, China; ^3^Department of General Surgery, Suzhou Hospital of Traditional Chinese Medicine, Suzhou 215000, China

## Abstract

**Aim:**

The aim of our work was to determine the utility of DNM1 as a biomarker for the diagnosis and prognosis of colon cancer (CC).

**Methods:**

DNM1 expression variations in CC vs. normal tissues were investigated using The Cancer Genome Atlas (TCGA) database. The association of DNM1 expression levels with the clinicopathological variables in CC prognosis was investigated using logistic regression analyses. Independent prognostic factors for CC were evaluated using univariate and multivariate Cox regression analyses. The correlation between DNM1 expression and immune cell infiltration was estimated using single-sample Gene Set Enrichment Analysis (ssGSEA).

**Results:**

DNM1 expression in CC tissues was significantly higher than that in normal tissues. High DNM1 expression was significantly correlated with M stage, N stage, perineural invasion and lymphatic invasion and predicted poor prognosis. The univariate analysis highlighted that DNM1 was an independent CC risk factor. Results of ssGSEA showed that DNM1 was linked to several cancer-related pathways, including the neuroactive ligand-receptor interaction, hypertrophic cardiomyopathy, ECM-receptor interaction, dilated cardiomyopathy, and calcium signaling pathway. Moreover, DNM1 expression was positively correlated with the level of infiltration by Neutrophils, Tregs, NK cells, and Macrophages.

**Conclusion:**

DNM1 has a significant function and has diagnostic and prognostic potential for CC.

## 1. Introduction

It is estimated that colon cancer (CC) is among the leading cancers globally. Annually, nearly 1.1 million new cases of CC and 551,000 CC deaths occur each year [1]. Colon adenocarcinoma (COAD) is the most common pathological type and accounts for >90% of CC cases [2]. The prognosis of CC always depends on the cancer stage at diagnosis. However, CC is often detected at an advanced stage, after lymph node and distant metastases occurred, resulting in poor overall survival [3]. Colonoscopy is the gold standard for diagnosing CC, but while highly sensitive, it is invasive and may cause serious complications [4, 5]. Additionally, due to high tumor heterogeneity at the single-cell level, local tumor biopsy results often fail to reflect the overall biology of the tumor and its disease process, which may contribute to the increased incidence of recurrence and metastases of CC [6, 7]. Although serum biomarkers like carbohydrate CA19-9 and CEA are commonly used in cancer diagnosis and prognosis, their sensitivity and specificity are not high [8]. Recently, several studies have pointed to the influence of the immune microenvironment on the development of colon cancer, suggesting that different types of immune cell infiltration may be used as new diagnostic and prognostic biomarkers [9, 10].

Dynamin is a 96 kDa GTPase, and the conventional dynamin family is composed of dynamins 1, 2, and 3 [11]. Of these, dynamin 1 (DNM1; NM_004408) is located on chromosome 9q34.11 and is expressed at different levels in various tissues, where it regulates cell membrane division, cytokinesis, and vesicle secretion [12]. DNM1 is often thought to be neuron-specific [13], and many studies have implicated it in neurological disorders [14–16]. However, recent studies have implicated DNM1 in the development of various cancers, such as bladder cancer (BC), non-small-cell lung cancer (NSCLC), and hepatocellular carcinoma (HCC) [17–19]. Therefore, the role of DNM1 in CC prognosis is unclear. Here, we investigated DNM1 expression in CC to determine its potential to be a useful biomarker for CC diagnosis and prognosis.

## 2. Materials and Methods

### 2.1. Data Collection and Analysis

COAD patients' RNA-Seq data and related clinical records were obtained from TCGA database (https://portal.gdc.cancer.gov) in March 2021 [20]. Upon excluding those lacking clinical information, 455 patients were included in our study. Based on the DNM1 expression level in tumor tissues, patients were classified into low- and high-expression groups.

### 2.2. Gene Set Enrichment Analysis (GSEA)

GSEA [21] is a genome-wide expression analysis tool that compares genes to a predefined gene collection. Based on the association of DNM1 expression with all genes, GSEA was conducted to create an organized list of genes for our analysis. Next, 1000 gene set alignments were executed for each analysis based on DNM1 levels as the phenotypic marker. Significant enrichment was considered for the normal *p* value < 0.05 and false discovery rate (FDR) < 0.25. Further, the normalized enrichment score (NES) and adjusted *p* value were employed to identify pathways enriched in each phenotype.

### 2.3. Immune Infiltration Analysis

Single-sample GSEA (ssGSEA) was used to determine the infiltration levels of tumor immune cells based on RNA-Seq data [22]. Spearman's correlation was used to examine the relationship between DNM1 and immune cells, and graphs were generated using ggplot2.

### 2.4. Statistical Analysis

TCGA RNA-Seq gene expression level 3 data and clinical information for all CC patients were analyzed on R version 3.6.3 [23], and *p* < 0.05 was considered statistically significant. Logistic regression (calculation of ORs and 95% CIs) and Wilcoxon signed-rank test were used to determine the correlation between DNM1 expression and CC clinicopathological features. The impact of DNM1 on the prognosis of COAD was evaluated using Kaplan-Meier and Cox regression analyses.

## 3. Results

### 3.1. Correlation between DNM1 Expression and Clinicopathological Features

The DNM1 level was substantially elevated in tumor samples than in normal samples (Figure 1(a), *p* < 0.0001). Similar results were found when comparing DNM1 expression in 41 pairs of patients (Figure 1(b), *p* < 0.0001). Wilcoxon signed-rank test analysis of the relationship between DNM1 expression and CC clinicopathological features showed that high DNM1 expression significantly correlated with higher N stage (Figure 2(e), *p* = 3.3∗10^−6^), higher M stage (Figure 2(f), *p* = 0.04), more perineural invasion (Figure 2(g), *p* = 0.01), and more lymphatic invasion (Figure 2(h), *p* = 6.4∗10^−5^). Similar results were obtained using chi-squared analysis of baseline patient data (Table 1). In the univariate logistic regression analysis, the DNM1 level was found strongly correlated with clinicopathological features (Table 2), including N stage (OR = 2.092, 95% CI: 1.445-3.042, and *p* < 0.001), M stage (OR = 1.885, 95% CI: 1.103-3.287, and *p* = 0.022), pathologic stage (OR = 2.033, 95% CI: 1.402-2.960, and *p* < 0.001), perineural invasion (OR = 2.744, 95% CI: 1.376-5.670, and *p* = 0.005), and lymphatic invasion (OR = 2.018, 95% CI: 1.364-3.001, and *p* < 0.001). However, DNM1 expression did not significantly correlate with age (OR = 1.190, 95% CI: 0.826-1.716, and *p* = 0.352), gender (OR = 1.106, 95% CI: 0.772-1.585, and *p* = 0.583), and T stage (OR = 1.311, 95% CI: 0.835-2.071, and *p* = 0.241). Together, these results suggest that high DNM1 expression predicts poor CC clinicopathological features.

### 3.2. High DNM1 Expression Affects Colon Cancer Prognosis

Relative to patients with low DNM1 levels, overall survival (OS) was significantly lower in those with high DNM1 levels (HR = 1.72, 95% CI: 1.16-2.56, and *p* = 0.007, Figure 3(a)). Similar results were obtained for disease-specific survival (DSS) (HR = 1.84, 95% CI: 1.11-3.06, and *p* = 0.006, Figure 3(b)) and progression-free interval (PFI) (HR = 1.74, 95% CI: 1.22-2.48, and *p* = 0.002, Figure 3(c)). Univariate analysis of CC prognostic factors revealed that age, T level, lymphatic invasion, M stage, N stage, pathologic stage, and high DNM1 expression are independent prognostic factors for CC (all *p* < 0.05). Multivariate Cox regression analysis showed that age, M stage, and pathologic stage were independent prognostic risk factors for OS in CC patients(all *p* < 0.05, Table 3).

### 3.3. GSEA Identifies DNM1-Related Signaling Pathways

KEGG pathway analysis identified differentially activated mechanisms and signaling pathways in CC from high DNM1-expression datasets from TCGA (FDR < 0.05, NOM *p* < 0.05). The results of GSEA showed that DNM1-related CC significantly correlated with tumorigenesis and involves various key pathways, including the calcium signaling pathway, dilated cardiomyopathy, neuroactive ligand-receptor interaction, hypertrophic cardiomyopathy (HCM), and ECM-receptor interaction (Figure 4, Table 4).

### 3.4. Correlation between DNM1 Levels and Immune Cell Infiltration Levels

Tumor-infiltrating lymphocytes can independently reflect cancer survival. Here, we examined if the DNM1 expression level correlated with infiltration of 24 immune cell subpopulations in CC [24] and found that DNM1 expression correlated with Neutrophils, Tregs, NK cells, and Macrophages. We also found a negative correlation between DNM1 levels and T helper cells, Th17 cells, and Th2 cells (Figure 5). Further analysis showed that DNM1 expression had a significant positive correlation with the infiltration level by Neutrophils (Figure 6(a), *r* = 0.3, *p* < 0.001), Tregs (Figure 6(b), *r* = 0.310, *p* < 0.001), NK cells (Figure 6(c), *r* = 0.35, *p* < 0.001), and Macrophages (Figure 6(d), *r* = 0.32, *p* < 0.001).

## 4. Discussion

Colon cancer has been a challenging clinical condition globally [1]. In recent years, the use of targeted therapies has greatly improved the OS of CC patients [25]. However, the global annual mortality rate remains high, further reinforcing the importance of discovering new biomarkers and using them for early diagnosis, prognosis, and treatment of CC. DNM1 belongs to the dynamin family [11], and numerous studies have implicated DNM1 in encephalopathy [14–16]. Additionally, recent studies indicated that DNM1 is highly expressed in tumor tissues and strongly correlated with cancer prognosis. Tian et al. [19] found that DNM1 was highly expressed in HCC tissues and DNM1 expression significantly correlated with the alpha-fetoprotein (AFP) level, T stage, and TNM stages in HCC. Besides, they found that high DNM1 expression also predicted poor OS in the HCC patients [19]. Schmid [26] recently found that clathrin-mediated endocytosis (CME) in H1299 NSCLC cells is Drp1- (dynamin-related protein 1-) dependent and sensitive to Akt inhibition, indicating its potential as a therapeutic target for NSCLC treatment. Chen et al. [27] showed that isoform-specific upregulation of clathrin light chain B and DNM1 in NSCLC cells, combined with the Akt/GSK3*β* signaling crosstalk, leads to clathrin-mediated adaptive endocytosis, which altered EGFR trafficking and NSCLC metastasis. Reis et al. [28] found that DNM1 overexpression selectively activates tumor necrosis factor- (TNF-) related apoptosis-inducing ligand death receptors to modulate endocytosis, suppress apoptosis, and improve cell migration and survival, indicating that reduced DNM1 expression may sensitize cells to apoptosis induction, while increased DNM1 expression levels may promote apoptosis resistance, thereby enhancing tumorigenesis and cancer progression. DNM1 is highly expressed in various cancers, including acute myeloid leukemia and lung cancer [29], probably due to its effect on apoptosis. Previous studies suggested that DNM1 has the potential to be a biomarker for cancer diagnosis, prognosis, and therapy. Our study showed that DNM1 was highly expressed in CC tissues relative to normal tissues, which also suggested that it may serve an essential role in CC development. Besides, we found high DNM1 expression closely correlated with the clinicopathological features of CC and predicted higher N stage, higher M stage, more peripheral invasion and lymphatic invasion. Similar results were obtained by chi-squared analysis of baseline patient data. Moreover, CC patients with higher DNM1 expression had worse OS, DSS, and PFI compared to those with low DNM1 expression. Univariate analysis showed that CC patients with advanced age, higher T stage, N stage, M stage, more advanced pathologic stage, lymphatic invasion, and higher DNM1 expression had significantly lower OS. However, multivariate Cox regression analysis confirmed that age, M stage, and pathologic stage were independent prognostic factors for CC.

To further investigate the function of DNM1 in CC, we performed GSEA on TCGA data, and the results showed that the calcium signaling pathway, ECM-receptor interaction, and neuroactive ligand-receptor interaction in KEGG are differentially enriched in the high DNM1-expression phenotype. Activation of the calcium signaling pathway promotes CC progression [30], suggesting regulation of this pathway as a new avenue for preventing CC development. Cell migration is a highly coordinated process involving the integration of ECM with the actin cytoskeleton across the plasma membrane via receptors [31]. Focal adhesion kinase (FAK) may be activated by the ECM, and its tyrosine phosphorylation facilitates the formation of focal complexes that mature into focal adhesions [32]. Wang et al. [33] found that targeted regulation of miR-17-5p may affect the neuroactive ligand-receptor interaction pathway and promote the proliferation and apoptosis of gastric cancer cells. CC immunotherapy studies have sought to identify new biomarkers and create rational combination therapy protocols. Thus, drugs targeting these signaling pathways may offer new therapeutic opportunities for CC therapy management.

The tumor microenvironment has a crucial role in tumorigenesis [34]. Our study of the correlation between DNM1 and immune cells found that neutrophils, Tregs, NK cells, and macrophages positively correlate with DNM1 expression, highlighting the importance of DNM1 in regulating the CC tumor immune microenvironment. Neutrophils, the main inflammatory component in tumors, produce cytokines and stimulate tumor progression [35]. Tumor-associated neutrophils (TANs) can recruit immune T cells, which may promote tumor growth, progression, and resistance to chemotherapy [36]. Zhang et al. [37] demonstrated that TANs can independently influence OS and DFS in colorectal cancer. Tregs reduce immunotherapy effectiveness due to their antitumor immune effects [38]. Thus, anti-Treg immunotherapy may be highly effective in CC patients. NK cells are natural lymphocytes that can kill viral infections or cancer cells [39]. Imai et al. [40] found that tumor progression was associated with reduced NK cells' killing capacity in peripheral blood. Thus, NK cells control tumorigenesis and hold great promise as an anti-CC immunotherapeutic target. Macrophages are critical components of the innate immune system [41], and tumor-associated macrophages (TAM) in the tumor microenvironment accelerate angiogenesis, immunosuppression, and cancer cell proliferation, thereby supporting tumor metastasis and growth [42]. Researchers have attempted to restore or enhance the killing ability of macrophages against tumor cells through various approaches, including inhibiting the transformation of TAM to the M1 type and promoting their activation as antigen-presenting cells against other antitumor effector cells, making macrophages an important member of tumor immunotherapy studies [43–45]. These findings suggest that the effect of DNM1 in CC may be significantly associated with immune infiltration. Our study is the first to clarify the influence of DNM1 expression on CC. Although our results have clinical significance, the study still has some limitations. Firstly, it lacks experimental validation. Secondly, data used in the study were obtained from TCGA only; thus, some biological information may be inevitably overlooked, leading to bias in the final results.

In summary, our findings suggest that high DNM1 expression closely correlates with poor CC prognosis. The key potential DNM1-regulated pathways in CC are neuroactive ligand-receptor interaction, hypertrophic cardiomyopathy (HCM), ECM-receptor interaction, calcium signaling, and dilated cardiomyopathy. Moreover, the DNM1 expression level significantly correlates with infiltration by neutrophils, Tregs, NK cells, and macrophages. Thus, DNM1 has the potential as a biomarker for the diagnosis and prognosis of colon cancer.

## Figures and Tables

**Figure 1:** (a) Relative to normal tissues, DNM1 expression was elevated in tumor tissues. (b) DNM1 was elevated in tumor tissues compared to normal ones in 41 paired patients.

**Figure 2:** Expression patterns of DNM1 in COAD from 478 RNA-Seq data. (a) Age at diagnosis. (b) Gender. (c) Pathologic stage. (d) T stage. (e) N stage. (f) M stage. (g) Perineural invasion. (h) Lymphatic invasion.

**Figure 3:** High DNM1 expression predicts poor prognosis of CC. (a) OS in CC patients with differential DNM1 expression (*p* = 0.007). (b) DSS in CC patients with differential DNM1 expression (*p* = 0.018). (c) PFI in CC patients with differential DNM1 expression (*p* = 0.002).

**Figure 4:** Enrichment gene set enrichment analysis (GSEA) plots. DNM1 was differentially enriched in the calcium signaling pathway, dilated cardiomyopathy, ECM-receptor interaction, hypertrophic cardiomyopathy (HCM), and neuroactive ligand-receptor interaction. There are no signaling pathways associated with low DNM1 expression based on the NES, NOM *p* value, and FDR value. ES: enrichment score; NES: normalized ES; FDR: false discovery rate.

**Figure 5:** Correlation analysis of DNM1 levels and immune cell infiltration.

**Figure 6:** Association analysis between the DNM1 expression and immune cell infiltration levels. (a) Neutrophils. (b) Tregs. (c) NK cells. (d) Macrophages.

**Table 1:** Correlation between DNM1 expression and CC clinicopathological features.

Characteristics	Low DNM1 expression	High DNM1 expression	*p*
*n*	239	239	
Age, *n* (%)			0.402
≤65	102 (21.3%)	92 (19.2%)	
>65	137 (28.7%)	147 (30.8%)	
Gender, *n* (%)			0.647
Female	116 (24.3%)	110 (23%)	
Male	123 (25.7%)	129 (27%)	
T stage, *n* (%)			0.540
T1	6 (1.3%)	5 (1%)	
T2	46 (9.6%)	37 (7.8%)	
T3	160 (33.5%)	163 (34.2%)	
T4	26 (5.5%)	34 (7.1%)	
N stage, *n* (%)			<0.001
N0	163 (34.1%)	121 (25.3%)	
N1	50 (10.5%)	58 (12.1%)	
N2	26 (5.4%)	60 (12.6%)	
M stage, *n* (%)			0.030
M0	181 (43.6%)	168 (40.5%)	
M1	24 (5.8%)	42 (10.1%)	
Pathologic stage, *n* (%)			0.002
Stage I	44 (9.4%)	37 (7.9%)	
Stage II	108 (23.1%)	79 (16.9%)	
Stage III	54 (11.6%)	79 (16.9%)	
Stage IV	24 (5.1%)	42 (9%)	
Perineural invasion, *n* (%)			0.007
No	77 (42.5%)	58 (32%)	
Yes	15 (8.3%)	31 (17.1%)	
Lymphatic invasion, *n* (%)			<0.001
No	149 (34.3%)	117 (27%)	
Yes	65 (15%)	103 (23.7%)	

**Table 2:** Logistic regression analysis of DNM1 expression associated with clinicopathological features.

Characteristics	Total (*n*)	Odds ratio (OR)	*p*
Age (>65 vs. ≤65)	478	1.190 (0.826-1.716)	0.352
Gender (male vs. female)	478	1.106 (0.772-1.585)	0.583
T stage (T3 & T4 vs. T1 & T2)	477	1.311 (0.835-2.071)	0.241
N stage (N1 & N2 vs. N0)	478	2.092 (1.445-3.042)	<0.001
M stage (M1 vs. M0)	415	1.885 (1.103-3.287)	0.022
Pathologic stage (Stage III & Stage IV vs. Stage I & Stage II)	467	2.033 (1.402-2.960)	<0.001
Perineural invasion (yes vs. no)	181	2.744 (1.376-5.670)	0.005
Lymphatic invasion (yes vs. no)	434	2.018 (1.364-3.001)	<0.001

**Table 3:** Univariate analysis and multivariate analysis of the correlation of DNM1 expression with OS among CC patients.

Characteristics	Total (*n*)	Univariate analysis		Multivariate analysis	
		Hazard ratio (95% CI)	*p*	Hazard ratio (95% CI)	*p*
Age (>65 vs. ≤65)	477	1.610 (1.052-2.463)	0.028	2.366 (1.011-5.536)	0.047
Gender (male vs. female)	477	1.101 (0.746-1.625)	0.627		
T stage (T3 & T4 vs. T1 & T2)	476	3.072 (1.423-6.631)	0.004	0.730 (0.134-3.986)	0.716
N stage (N1 & N2 vs. N0)	477	2.592 (1.743-3.855)	<0.001	0.153 (0.014-1.609)	0.118
M stage (M1 vs. M0)	414	4.193 (2.683-6.554)	<0.001	3.022 (1.158-7.887)	0.024
Pathologic stage (Stage III & Stage IV vs. Stage I & Stage II)	466	2.947 (1.942-4.471)	<0.001	17.160 (1.348-218.491)	0.029
Perineural invasion (yes vs. no)	181	1.940 (0.982-3.832)	0.056	0.979 (0.388-2.470)	0.964
Lymphatic invasion (yes vs. no)	433	2.450 (1.614-3.720)	<0.001	1.318 (0.512-3.392)	0.567
DNM1 (high vs. low)	477	1.725 (1.163-2.558)	0.007	2.370 (0.859-6.536)	0.096

**Table 4:** Enrichment plots for gene set enrichment analysis (GSEA).

Description	Set size	Enrichment score	NES	*p* value	*p*.adjust	*q* values	Rank	leading_edge
KEGG_CALCIUM_SIGNALING_PATHWAY	177	0.5413707	1.39626282	0.000999	0.03299416	0.02839298	9738	Tags = 50%, list = 27%, signal = 37%
KEGG_DILATED_CARDIOMYOPATHY	90	0.57422622	1.45061151	0.000999	0.03299416	0.02839298	9738	Tags = 53%, list = 27%, signal = 39%
KEGG_ECM_RECEPTOR_INTERACTION	83	0.60605187	1.52489243	0.000999	0.03299416	0.02839298	7196	Tags = 53%, list = 20%, signal = 43%
KEGG_HYPERTROPHIC_CARDIOMYOPATHY_HCM	83	0.57650225	1.45054239	0.000999	0.03299416	0.02839298	9738	Tags = 52%, list = 27%, signal = 38%
KEGG_NEUROACTIVE_LIGAND_RECEPTOR_INTERACTION	270	0.58383597	1.51792562	0.000999	0.03299416	0.02839298	8274	Tags = 55%, list = 23%, signal = 43%

## Data Availability

Publicly available datasets were analyzed in this study. These data can be found here: https://portal.gdc.cancer.gov. The data from TCGA are publicly available and open-access. Therefore, the local ethics committees did not need to approve the study because the current research follows TCGA data access policies and publication guidelines.
